The article "Effect of Early Enteral Nutrition Support Combined with Chemotherapy on Related Complications and Immune Function of Patients after Radical Gastrectomy" was published in 2022. Journal: J Healthc Eng.

# Effect of Early Enteral Nutrition Support Combined with Chemotherapy on Related Complications and Immune Function of Patients after Radical Gastrectomy

**DOI:** 10.1155/2022/1531738

**Published:** 2022-01-27

**Authors:** Jing Wang, Lei Wang, Min Zhao, Xiaoxia Zuo, Wenhua Zhu, Keying Cui, Xu Yan, Xiaofei Liu

**Affiliations:** ^1^Department of Clinical Nutrition, The 8th Medical Center of Chinese PLA General Hospital, Beijing 100091, China; ^2^Department of Clinical Nutrition, The First Affiliated Hospital, Zhejiang University School of Medicine, Hangzhou 310003, Zhejiang Province, China; ^3^Department of Clinical Nutrition, The 6th Medical Center of Chinese PLA General Hospital, Beijing 100048, China; ^4^Department of Oncology, The 8th Medical Center of Chinese PLA General Hospital, Beijing 100091, China; ^5^Department of General Surgery, The 8th Medical Center of Chinese PLA General Hospital, Beijing 100091, China; ^6^Department of Nuclear Medicine, The 8th Medical Center of Chinese PLA General Hospital, Beijing 100091, China

## Abstract

**Objective:**

The purpose was to analyze the effect of early enteral nutrition (EEN) support combined with chemotherapy on related complications and immune function in patients after radical gastrectomy.

**Methods:**

80 patients with gastric cancer treated in our hospital from March 2019 to March 2020 were selected as the research objects and divided into the experimental group and control group according to the random number table, with 40 cases in each group. The control group received chemotherapy only after surgery, while the experimental group received EEN on this basis. The total protein (TP), transferrin (TF), albumin (ALB), immune cells, and other indexes were measured in the two groups before and after treatment to analyze the effect of different treatment methods on the complications and immune function of patients after radical gastrectomy.

**Results:**

There were no significant differences in gender ratio, average age, average BMI, pathological types, disease staging, and residence between the two groups (*P* > 0.05). The exhaust recovery time, total gastric tube drainage, fluid intake time, and hospitalization time in the experimental group were significantly lower than those in the control group (*P* < 0.05). There were no significant differences in the TP, TF, and ALB levels between the two groups before treatment (*P* > 0.05), and the TP, TF, and ALB levels in the experimental group were significantly higher than those in the control group after treatment (*P* < 0.05). The CD4^+^/CD8^+^, CD3^+^, and CD4^+^ levels in the experimental group after treatment were significantly higher than those in the control group (*P* < 0.001). After treatment, the growth hormone levels in both groups significantly increased (*P* < 0.001), and the growth hormone level in the experimental group was significantly higher than that in the control group (*P* < 0.001). There was no significant difference in the KPS scores between the two groups before treatment (*P* > 0.05), and the KPS score in the experimental group was significantly higher than that in the control group after treatment (*P* < 0.001). The incidence of postoperative complications in the experimental group was significantly lower than that in the control group (*P* < 0.05).

**Conclusion:**

EEN combined with chemotherapy is a reliable method to improve the immune function of patients after radical gastrectomy for gastric cancer, which plays an important role in improving the physical state of patients and reducing the incidence of complications. Therefore, its further research will help to establish a better treatment plan for such patients.

## 1. Introduction

Gastric cancer is a common digestive tract malignant tumor disease with a high incidence worldwide [1]. Radical gastrectomy is currently the preferred treatment method for gastric cancer. However, different damage to the gastrointestinal and immune functions of patients will occur under the influence of surgery and tumor consumption, resulting in malnutrition. In addition, gastric cancer patients often need adjuvant chemotherapy after surgery, but the adverse reactions caused by chemotherapy will affect the treatment compliance of patients to a certain extent, increasing the treatment pain and affecting the gastrointestinal function [2–4]. Impaired gastrointestinal absorption function can affect the intake of nutrients, reduce immunity, increase the risk of postoperative infection, and affect prognosis. Therefore, how to improve the gastrointestinal and immune functions of patients after surgery and timely correct malnutrition has become an urgent problem for doctors. EEN has gained extensive concern because studies have confirmed that EEN can effectively reduce the nutritional intake of patients after surgery. However, there is no unified understanding of the effect of EEN on the related complications and immune function of patients after radical gastrectomy [5]. Based on this, this study aims to further explore the effect of EEN support combined with chemotherapy on related complications and immune function of patients after radical gastrectomy and provide a basis for clinical applications, summarized as follows.

## 2. Materials and Methods

### 2.1. General Information

80 patients with gastric cancer treated in our hospital from March 2019 to March 2020 were selected as the research objects and divided into the experimental group and control group according to the random number table, with 40 cases in each group. The study was conducted in accordance with the Declaration of Helsinki (as revised in 2013) [6].

### 2.2. Inclusion Criteria

The inclusion criteria were as follows: ① the patients were diagnosed with gastric cancer after imaging examinations such as gastroscopy and CT and confirmed by histopathological examination, with the clinical symptoms such as fatigue, anorexia, upper abdominal pain, hematemesis, and melena; ② the patients received radical gastrectomy (distal gastrectomy, total gastrectomy, and proximal gastrectomy) and had normal intestinal function before surgery; and ③ the patients did not take immunosuppressants recently.

### 2.3. Exclusion Criteria

The exclusion criteria were as follows: ① the patients were complicated with immunodeficiency, liver and kidney dysfunction, and endocrine diseases before surgery; ② the patients received parenteral or enteral nutrition treatment, accompanied by severe gastrointestinal dysfunction; ③ the patients had tumor distant metastasis; and ④ the patients were allergic to nutrient solution.

### 2.4. Methods

Patients in the control group received chemotherapy after surgery, including tetrahydrofolic acid, oxaliplatin, and fluorouracil. 400 mg/m^2^ of tetrahydrofolate acid (SFDA approval no. H15021455; manufacturer: Chifeng Mengxin Pharmaceutical Co., Ltd.; specification: 15 mg/s) was intravenously injected to the patients on the 1st day. Oxaliplatin (SFDA approval no. H20143023; manufacturer: Hainan Jinrui Pharmaceutical Co., Ltd.; specification: 50 mg) was intravenously injected on the 1st day, with 85 mg/m^2^ dripping for more than 2 hours. Fluorouracil injection (manufacturer: Shanghai Xudong Haipu Pharmaceutical Co., Ltd.; NMPA approval no. H31020593; specification: 10 ml: 0.25 g) was injected on the 2nd day, with a single dose of 10–20 mg/kg each day according to the patients' body weight and 2 weeks as a cycle.

The experimental group received EEN support based on the treatment of the control group. The nasointestinal tube was placed at 30–40 cm below the jejunal anastomosis, and 0.9% and 500 ml NaCl solution was infused in 12–24 hours after surgery. Enteral nutritional emulsion (TP) was infused to the patients at 24 hours after surgery, with the calorie as 30 mL (30 kcaD/kg·d) and the nutritional components including saturated fatty acid (1.6%), fat (3.4%), protein (3.8%), unsaturated fatty acid (1.3%), carbohydrate (13.8%), medium-chain triglyceride (1.2%), and sugar (0.5%). The emulsion was continuously infused for 7 days, following the principle of “first slow and then fast, and first dilute and then thick.” The dosage and infusion rate were gradually adjusted according to the patients' tolerance, from half amount to full amount. After oral diet, patients could gradually reduce the intake of enteral nutrition and properly supplement electrolytes, vitamins, and trace elements. The temperature of nutrient solution was controlled at about 39°C to avoid cold stimulation which caused intestinal spasm, leading to abdominal pain and diarrhea [7, 8].

### 2.5. Observation Indexes

The exhaust recovery time, total gastric tube drainage, fluid intake time, and hospitalization time were recorded and compared between the two groups.

5 ml of fasting venous blood was collected from both groups before and after treatment, and the upper serum was taken after centrifugation. An automatic biochemical analyzer (manufacturer: Beijing Perlong Technology Co., Ltd.; model: 600A/B) was used to detect the nutritive indexes (TP, TF, and ALB) in both groups before and after treatment.

A flow cytometer (manufacturer: Shanghai Huanxi Medical Devices Co., Ltd.; model: XTG-1600E) was used to detect the CD3^+^, CD4^+^, and CD4^+^/CD8^+^ levels.

Radioimmunoassay was used to detect the growth hormone level in both groups after treatment. The kits were purchased from Shanghai Hengyuan Biotechnology Co., Ltd.

Karnofsky score (KPS) [9] was used to evaluate the physical state in both groups before and after treatment. The total score of the scale was 100 points, and the score ≥80 indicated that the patients could completely take care of themselves, 50–79 indicated that the patients could partially take care of themselves, and ≤49 indicated that the patients could not take care of themselves.

The incidence of clinical complications during treatment was recorded and compared between the two groups, including diarrhea, abdominal pain, and phlebitis.

### 2.6. Statistical Methods

All the experimental data were statistically analyzed and processed by SPSS 21.0 software, and GraphPad Prism 7 (GraphPad Software, San Diego, USA) was used to draw pictures of the data. The count data were tested by *X*^2^, expressed by *n* (%), and the measurement data were measured by *t*-test, expressed by (‾*x* ± *s*). The difference was statistically significant when *P* < 0.05.

## 3. Results

### 3.1. Comparison of Baseline Data between the Two Groups

There were no significant differences in gender ratio, average age, average BMI, pathological types, disease staging, and residence between the two groups (*P* > 0.05), indicating comparability, as shown in Table 1.

### 3.2. Comparison of Postoperative Recovery between the Two Groups

The exhaust recovery time, total gastric tube drainage, fluid intake time, and hospitalization time in the experimental group were significantly lower than those in the control group (*P* < 0.05), as shown in Table 2.

### 3.3. Comparison of Nutritive Indexes before and after Treatment between the Two Groups

There were no significant differences in the TP, TF, and ALB levels between the two groups before treatment (*P* > 0.05), and the TP, TF, and ALB levels in the experimental group were significantly higher than those in the control group after treatment (*P* < 0.05), as shown in Table 3.

### 3.4. Comparison of Immune Indexes after Treatment between the Two Groups

The CD4^+^/CD8^+^, CD3^+^, and CD4^+^ levels in the experimental group after treatment were significantly higher than those in the control group (*P* < 0.05), as shown in Table 4.

### 3.5. Comparison of Growth Hormone Levels before and after Treatment between the Two Groups

After treatment, the growth hormone levels in both groups significantly increased (*P* < 0.05), and the growth hormone level in the experimental group was significantly higher than that in the control group (*P* < 0.05), as shown in Figure 1.

### 3.6. Comparison of KPS Scores before and after Treatment between the Two Groups

There was no significant difference in the KPS scores between the two groups before treatment (*P* > 0.05), and the KPS score in the experimental group was significantly higher than that in the control group after treatment (*P* < 0.05), as shown in Figure 2.

### 3.7. Comparison of the Incidence of Complications between the Two Groups

The incidence of postoperative complications in the experimental group was significantly lower than that in the control group (*P* < 0.05), as shown in Table 5.

## 4. Discussion

Gastric cancer can occur in any part of the stomach. The pathogenesis is that the mutation of a single gene results in the exponential growth of gastric cancer cells and decreased body's immune function or immune escape effect of gastric cancer cells so that the body's immune system cannot kill gastric cancer cells. At this time, cancer cells will break through the basal layer, and distant metastasis occurs through the lymphatic and blood systems, thereby affecting the normal diet and digestion and hindering the absorption of nutrients. Radical gastrectomy will cause stress reactions in patients, which accelerate the catabolism and aggravate the degree of malnutrition, leading to decreased immune function, postoperative complications, and poor prognosis [10–12]. Chemotherapy is a common auxiliary method for patients with gastric cancer after surgery, which can inhibit the subclinical disease in patients to a certain extent, reduce the activity of tumor cells, minimize the chance of tumor cell proliferation after surgery, and reduce the possibility of recurrence. In addition, chemotherapy can also reduce the adhesion of tumor tissue, decrease the clinical tumor stages, and improve the success rate of surgical resection [13–15]. However, chemotherapy will have severe strong gastrointestinal reactions, myelosuppression, alopecia, and other complications, increasing the pain of treatment and seriously affecting the life quality [16]. In addition, investigations have found that most patients with gastric cancer have varying degrees of malnutrition and immunosenescence symptoms before admission due to vomiting, tumor consumption, and other factors, which will further deteriorate after a series of clinical treatments such as surgery and chemotherapy. Therefore, how to implement nutritional support and treatment for patients after radical surgery is crucial to their rehabilitation, the improvement of immune function, and the reduction of related complications [17–19].

EEN can not only provide nutrition for patients but also reduce oxidative stress, protect the gastrointestinal structure and function, and reduce inflammatory response, so as to maintain the functions of organs, tissues, and cells, improve nutrition absorption rate, enhance immune function, and promote rehabilitation, which has been confirmed in diseases such as ischemic stroke, acute pancreatitis, and esophagus cancer [20, 21]. In this study, the patients in the experimental group received nutritional support with a nasointestinal tube which is simple and safe, with little impact on the patient comfort. In addition, the anastomotic stoma was avoided during feeding to avoid the food stimulation to the stoma and improve the nutritional absorption. After treatment, the exhaust recovery time, total gastric tube drainage, fluid intake time, and hospitalization time in the experimental group were significantly lower than those in the control group (*P* < 0.001), indicating that EEN combined with chemotherapy can significantly shorten the recovery time of patients after surgery, which is more effective than chemotherapy alone. The immune function is mainly exerted through cellular immunity, in which T lymphocytes are the main effector cells and can directly reflect the body immune condition in the perioperative period [22, 23]. EEN contributes to the recovery of intestinal function and maintains the integrity of the intestinal mucosal structure and function. This study showed that the CD4^+^/CD8^+^, CD3^+^, and CD4^+^ levels in the experimental group after treatment were significantly higher than those in the control group (*P* < 0.001). Tai et al. [24] pointed out that, after the patients with stage II gastric cancer received EEN based on the radical gastrectomy, the CD3^+^ and CD4^+^ levels of patients were 62.47 ± 3.64% and 42.18 ± 3.81%, which were significantly higher than 58.62 ± 3.49% and 36.34 ± 3.24% before treatment, suggesting that EEN can significantly improve the immune function of patients with gastric cancer after radical gastrectomy. In addition, the study also found that the incidence of postoperative complications in the experimental group was significantly lower than that in the control group (*P* < 0.05). It was speculated that EEN preparations were rich in nutrients such as fat, amino acids, and vitamins, which could enhance the blood flow in the gastrointestinal tract of patients, promote digestive movement and the secretion of related hormones, and provide the body with the required energy supply, thus improving the patients' own immunity and greatly reducing the risk of postoperative complications. Since this study is a single-center and small-sample test, it is not sufficient to assess the differences in postoperative immune function and complications. In order to reduce bias, the selected patients were screened, and those with endocrine diseases and distant metastasis of tumors were excluded. Therefore, this experiment cannot comprehensively describe the clinical symptoms of patients, but indicated the direction for the subsequent research studies.

In conclusion, EEN combined with chemotherapy is a reliable method to improve the nutritional status and immune function of patients with gastric cancer after radical gastrectomy. This treatment method greatly shortens the postoperative recovery time of patients and reduces the incidence of postoperative complications, which has a high clinical application value.

## Figures and Tables

**Figure 1:** Comparison of growth hormone levels before and after treatment between the two groups (‾*x* ± *s*). Note: the abscissa represents before treatment and after treatment, and the ordinate represents the growth hormone level (ng/L). The growth hormone levels in the experimental group before and after treatment were 94.25 ± 5.84 ng/L and 142.37 ± 6.94 ng/L, respectively. The growth hormone levels in the control group before and after treatment were 94.46 ± 5.69 ng/L and 123.54 ± 6.53 ng/L, respectively. ^*∗*^A significant difference in the growth hormone levels of the experimental group before and after treatment (*t* = 33.553, *P* < 0.001). ^*∗∗*^A significant difference in the growth hormone levels of the control group before and after treatment (*t* = 21.235, *P* < 0.001). ^*∗∗∗*^A significant difference in the growth hormone levels between the two groups after treatment (*t* = 12.498, *P* < 0.001).

**Figure 2:** Comparison of KPS scores before and after treatment between the two groups (‾*x* ± *s*). Note: the abscissa represents before treatment and after treatment, and the ordinate represents the KPS score (points). The KPS scores in the experimental group before and after treatment were 61.83 ± 3.54 and 72.42 ± 3.44, respectively. The KPS scores in the control group before and after treatment were 61.79 ± 3.63 and 65.96 ± 3.81, respectively.^*∗*^A significant difference in the KPS scores between the two groups after treatment (*t* = 7.959, *P* < 0.001).

**Table 1:** Comparison of baseline data between the two groups.

Items	Experimental group (*n* = 40)	Control group (*n* = 40)	*χ* ^2^/*t*	*P*
Gender			0.205	0.651
Male	22 (59.46%)	24 (64.86%)		
Female	18 (48.65%)	16 (43.24%)		
Average age (years)	43.71 ± 4.32	43.59 ± 4.36	0.124	0.902
Average BMI (kg/m^2^)	21.65 ± 1.26	21.57 ± 1.28	0.282	0.779
Pathological types				
Mucinous carcinoma	4 (10.00%)	6 (15.00%)	0.457	0.499
Medium differentiated adenocarcinoma	13 (32.50%)	12 (30.00%)	0.058	0.809
Poorly differentiated adenocarcinoma	6 (15.00%)	8 (20.00%)	0.346	0.556
Highly differentiated adenocarcinoma	17 (42.50%)	14 (35.00%)	0.474	0.491
Disease staging				
I	11 (27.50%)	13 (32.50%)	0.238	0.626
II	17 (42.50%)	14 (35.00%)	0.474	0.491
III	12 (30.00%)	13 (32.50%)	0.058	0.809
Residence			0.802	0.370
Urban area	19 (47.50%)	23 (57.50%)		
Rural area	21 (52.50%)	17 (42.50%)		

**Table 2:** Comparison of postoperative recovery between the two groups (‾*x* ± *s*).

Group	*n*	Exhaust recovery time (h)	Total gastric tube drainage (mL)	Fluid intake time (d)	Hospitalization time (d)
Experimental group	40	81.94 ± 13.27	263.81 ± 38.92	5.42 ± 1.06	12.52 ± 4.82
Control group	40	91.72 ± 12.65	374.81 ± 36.57	7.32 ± 1.21	17.24 ± 4.34
*t*		3.374	13.145	7.470	4.603
*P*		<0.05	<0.001	<0.001	<0.001

**Table 3:** Comparison of nutritive indexes before and after treatment between the two groups (‾*x* ± *s*).

Group	*n*	TP (g·L^−1^)		TF (mg·L^−1^)		ALB (g/L)	
		Before treatment	After treatment	Before treatment	After treatment	Before treatment	After treatment
Experimental group	40	58.21 ± 6.25	66.87 ± 5.82	127.69 ± 8.48	153.27 ± 6.79	26.51 ± 2.31	40.26 ± 3.18
Control group	40	58.27 ± 6.34	63.18 ± 5.42	127.73 ± 8.53	146.72 ± 6.54	26.47 ± 2.36	34.52 ± 3.14
*t*		0.043	2.934	0.021	4.394	0.077	8.123
*P*		0.966	<0.05	0.983	<0.001	0.939	<0.001

**Table 4:** Comparison of immune indexes after treatment between the two groups (‾*x* ± *s*).

Group	*n*	CD4^+^/CD8^+^	CD3^+^ (%)	CD4^+^ (%)
Experimental group	40	1.65 ± 0.42	64.32 ± 4.29	43.18 ± 3.19
Control group	40	1.32 ± 0.34	58.63 ± 4.38	38.71 ± 3.85
*t*		3.862	5.870	5.654
*P*		<0.001	<0.001	<0.001

**Table 5:** Comparison of the incidence of complications between the two groups (*n* (%)).

Group	*n*	Diarrhea	Abdominal pain	Phlebitis	Total incidence
Experimental group	40	2 (5.00%)	1 (2.50%)	1 (2.50%)	10.00% (4/40)
Control group	40	4 (10.00%)	4 (10.00%)	3 (7.50%)	27.50% (11/40)
*X* ^2^					4.021
*P*					<0.05

## Data Availability

The data used to support the findings of this study are available from the corresponding author upon reasonable request.
